The article "Synthesis, Characterization and In Vitro Study of Biocompatible Cinnamaldehyde Functionalized Magnetite Nanoparticles (CPGF Nps) For Hyperthermia and Drug Delivery Applications in Breast Cancer" was retracted in 2023. Reasons: concerns about the data; concerns about the results or conclusions.

# Synthesis, Characterization and In Vitro Study of Biocompatible Cinnamaldehyde Functionalized Magnetite Nanoparticles (CPGF Nps) For Hyperthermia and Drug Delivery Applications in Breast Cancer

**DOI:** 10.1371/journal.pone.0107315

**Published:** 2014-09-30

**Authors:** Kirtee D. Wani, Brijesh S. Kadu, Prakash Mansara, Preeti Gupta, Avinash V. Deore, Rajeev C. Chikate, Pankaj Poddar, Sanjay D. Dhole, Ruchika Kaul-Ghanekar

**Affiliations:** 1 Cell and Translational Research Laboratory, Interactive Research School for Health Affairs (IRSHA), Bharati Vidyapeeth University Medical College Campus, Dhankawadi, Pune, Maharashtra, India; 2 Nanoscience Group, Department of Chemistry, Post-graduate and Research Center, MES Abasaheb Garware College, Pune, Maharashtra, India; 3 Physical and Material Chemistry Division, CSIR-National Chemical Laboratory, Pune, Maharashtra, India; 4 Department of Physics, University of Pune, Pune, Maharashtra, India; Cedars-Sinai Medical Center; UCLA School of Medicine, United States of America

## Abstract

Cinnamaldehyde, the bioactive component of the spice cinnamon, and its derivatives have been shown to possess anti-cancer activity against various cancer cell lines. However, its hydrophobic nature invites attention for efficient drug delivery systems that would enhance the bioavailability of cinnamaldehyde without affecting its bioactivity. Here, we report the synthesis of stable aqueous suspension of cinnamaldehyde tagged Fe_3_O_4_ nanoparticles capped with glycine and pluronic polymer (CPGF NPs) for their potential application in drug delivery and hyperthermia in breast cancer. The monodispersed superparamagnetic NPs had an average particulate size of ∼20 nm. TGA data revealed the drug payload of ∼18%. Compared to the free cinnamaldehyde, CPGF NPs reduced the viability of breast cancer cell lines, MCF7 and MDAMB231, at lower doses of cinnamaldehyde suggesting its increased bioavailability and in turn its therapeutic efficacy in the cells. Interestingly, the NPs were non-toxic to the non-cancerous HEK293 and MCF10A cell lines compared to the free cinnamaldehyde. The novelty of CPGF nanoparticulate system was that it could induce cytotoxicity in both ER/PR positive/Her2 negative (MCF7) and ER/PR negative/Her2 negative (MDAMB231) breast cancer cells, the latter being insensitive to most of the chemotherapeutic drugs. The NPs decreased the growth of the breast cancer cells in a dose-dependent manner and altered their migration through reduction in MMP-2 expression. CPGF NPs also decreased the expression of VEGF, an important oncomarker of tumor angiogenesis. They induced apoptosis in breast cancer cells through loss of mitochondrial membrane potential and activation of caspase-3. Interestingly, upon exposure to the radiofrequency waves, the NPs heated up to 41.6°C within 1 min, suggesting their promise as a magnetic hyperthermia agent. All these findings indicate that CPGF NPs prove to be potential nano-chemotherapeutic agents in breast cancer.

## Introduction

Breast cancer is the second leading cause of cancer death in women worldwide [1]. The current treatment methods for breast cancer include chemotherapy, radiotherapy, and hormone therapy, which are used alone or in combination [2]. Despite advanced research in diagnostics and therapeutics, the associated side effects [3] as well as the recurrence [4] remain a few inevitable challenges in breast cancer therapy.

Recently, lot of research is being focussed towards the use of herbal medicines to minimize the side effects associated with conventional cancer therapy [5]. Medicinal plants are the valuable sources of anti-cancer bioactives such as curcumin, vinblastine, vincristine, paclitaxel, cinnamaldehyde, capsaicin, wogonin, berberine, artemisinin and so on, which have been shown to suppress and/or prevent cancer [6], [7]. However, most of these compounds are hydrophobic in nature and thus show decreased bioavailability [8]. This could be overcome by conjugating these herbal bioactives with biocompatible drug delivery agents that would improve their therapeutic efficacy [9], [10].

Cinnamaldehyde, a major bioactive component of the spice cinnamon has been reported to exhibit diverse biological functions including anticancer activity [11], [12], [13] (Table S1 in File S1). We have also previously reported the anticancer activity of cinnamaldehyde, however, at higher doses [12]. The therapeutic efficacy of cinnamaldehyde is limited due to its low water solubility [14]. This calls attention for drug delivery systems that would not only enhance the drug bioavailability without affecting its bioactivity but would also help in the targeted delivery of cinnamaldehyde at a lower dose.

The superparamagnetic nanoparticles (Fe_3_O_4_ MNPs) represent one of the most promising biocompatible nanomaterials that can be guided under an external magnetic field for magnetotherapy [15]. Magnetite nanoparticles (Fe_3_O_4_) have been loaded with different anticancer drugs including doxorubicin, daunorubicin, 5-bromotetrandrine [16], [17], [18], anti-HER2 immunoliposomes [19] and so on to evaluate their therapeutic potential in breast cancer. MNPs have also been loaded with natural herbal bioactives such as artesunate, silibinin, gambogic acid, tetrandrine, wogonin, curcumin, gallic acid and genistein; and studied for their anticancer efficacy as well as enhancement of bioavailability in cancer cells (Table S2 in File S1). Such studies reveal that the tagged bioactives possess enhanced efficacy than the free drug in terms of MIC and IC_50_ values. MNPs have been widely used for the drug delivery of anticancer agents because of their target specificity and sustained-release properties [15]. The property of target orientation of MNPs helps to reduce the systemic toxicity induced by the chemotherapeutic drugs [20].

In the present report, we have tagged cinnamaldehyde with Fe_3_O_4_ NPs that had been previously capped with glycine and pluronic polymer (CPGF NPs) to increase its therapeutic efficacy in breast cancer cells. CPGF NPs were initially characterized for their size, morphology, bonding properties and magnetism. They were analyzed for their drug loading and release profiles, stability and biocompatibility. CPGF NPs induced cytotoxicity in breast cancer cell lines at lower doses of cinnamaldehyde compared to the free cinnamaldehyde, thereby showing increased bioavailability in the cells. They also altered the growth kinetics of the cancer cells in a dose-dependent manner. The NPs reduced the migration capability of the cancer cells through reduction in the expression of MMP-2 along with decrease in a pro-angiogenesis marker, VEGF. The NPs also induced apoptosis in breast cancer cells through loss of mitochondrial membrane potential and increase in caspase-3 expression. Moreover, the RF studies indicated the potential of CPGF NPs in hyperthermia applications as well.

## Materials and Methods

### Chemicals and materials

The chemicals for synthesis, FeSO_4_.7H_2_O, Fe(NO_3_)_3_, NH_4_OH, glycine and pluronic F-127, were procured from Merck. Dulbecco's Modified Eagle's Medium (DMEM), penicillin/streptomycin and L-glutamine were obtained from Gibco BRL, CA, USA. Cinnamaldehyde, foetal bovine serum (FBS), 3-(4, 5-dimethylthiazol-2-yl)-2, 5-diphenylthiazolium bromide (MTT), FCCP and JC-1 were procured from Sigma-Aldrich (St. Louis, MO, USA). Neutral red and potassium ferrocyanide were obtained from Sd Fine-Chem. Ltd. Mumbai, India. Antibodies against caspase-3, VEGF and α-tubulin were purchased from Santa Cruz Biotechnology, Inc. (Santa Cruz, CA, USA). All other common reagents were procured from Qualigens fine chemicals (Mumbai, India).

### Cell culture

Tissue culture plasticware was purchased from BD Biosciences (CA, USA). MDAMB231, MCF7, MCF10A and HEK 293 were obtained from National Centre for Cell Science (NCCS), Pune. The cells were grown in DMEM supplemented with 2 mM L-glutamine, 100 units/ml of penicillin/streptomycin, and 10% fetal bovine serum (FBS). They were incubated in a humidified 5% CO_2_ incubator at 37°C.

### Synthesis of iron oxide (F), glycine capped (GF), Glycine and Pluronic stabilized (PGF) and cinnamaldehyde tagged (CPGF) NPs

#### 1. Iron oxide (F) nanoparticle synthesis

Pure iron oxide nanoparticles were synthesized by co-precipitation of ferric and ferrous salts in oxygen free atmosphere at ambient temperature [21]. 100 ml of water containing FeSO_4_.7H_2_O (0.556 g, 1 mM) and Fe(NO_3_)_3_ (1.636 g, 2 mM) (1∶2 molar ratio) was magnetically stirred at 800 rpm under N_2_ protection at 80°C for 20 min into a three-necked, round-bottomed flask in a rotamantle (Remi, India). To this solution, 50 ml of 30% ammonia was added slowly by a drop funnel and the speed was increased to 1200 rpm in order to uniformly precipitate magnetic nanoparticles. The colour of the suspension immediately turned black, indicating the formation of magnetite. The resulting solution was stirred for another 20 min followed by rapid cooling to room temperature using an ice bath to prevent further particle growth. The resulting black precipitate was collected with a strong magnet and the supernatant was removed from the precipitate by decantation. The slurry was washed four times with distilled water (DW) to remove excess ammonia and was monitored by a pH drop from 10 to 7. The nanoparticles were re-suspended in 25 ml water and centrifuged at 1000 rpm to remove larger aggregates. These F NPs were characterized and used for biological experiments.

#### 2. Glycine capped iron oxide (GF) nanoparticle synthesis

Similar to the method described above, glycine capped iron oxide nanoparticles were synthesized by co-precipitation of FeSO_4_.7H_2_O (0.556 g, 1 mM), Fe(NO_3_)_3_ (1.636 g, 2 mM) (1∶2 molar ratio) along with glycine (3 g, 0.4 M). The synthesis method and conditions were same as that for bare iron oxide nanoparticles. These GF NPs were characterized and used for biological experiments.

#### 3. Glycine capped pluronic stabilized iron oxide (PGF) nanoparticle synthesis

GF NPs were further coated with pluronic by adding 500 mg pluronic to get a thin coating. The mixture containing FeSO_4_.7H_2_O, Fe(NO_3_)_3_, glycine, ammonia and pluronic was stirred for another 20 min followed by rapid cooling. NPs were washed with DW as described earlier. To ensure complete coating of glycine and pluronic over the nanoparticles, the slurry obtained above was further subjected to sonication for 5 min followed by stirring for 1 h. The NPs were re-suspended in 25 ml water and centrifuged at 1000 rpm to remove larger aggregates. These PGF NPs were characterized and used for biological experiments.

#### 4. Cinnamaldehyde tagged iron oxide (CPGF) nanoparticle synthesis

Briefly, PGF NPs were suspended in 25 ml of absolute ethanol. To this mixture, 0.1 M cinnamaldehyde in 1 ml of ethanol was added and then it was vortexed for 1 h. The solution was magnetically stirred overnight at 900 rpm to complete the reaction. After the magnetic separation, the particles were re-suspended in different grades of ethanol (100%, 70%, 50%) and finally in 25 ml DW. The suspension was centrifuged at 1000 rpm to remove larger aggregates. The final CPGF NPs were used for either biological experiments or were vacuum dried to fine powder that was used for physical characterization.

### Physical characterization

The magnetic nanoparticles (F, GF, PGF and CPGF) were vacuum dried to obtain fine powder and used for the physical characterization by X-ray diffraction (XRD), Fourier transform infrared (FTIR) spectroscopy, thermo-gravimetric analysis (TGA), and vibrating sample magnetometry (VSM). Determination of phase purity and identification of NPs was done by XRD using powder diffractometer (Shimadzu, Physics Department, Pune University, Pune) with Cu radiation, operating at 40 kV and 40 mA. For TEM analysis, the colloidal solutions of NPs were ultrasonicated for 15 min. Bonding patterns of all the NPs were studied by FTIR (Shimadzu IR Infinity, Physics department, Pune University, Pune) and the data was acquired between 4000 and 400 cm^−1^. Percentage of cinnamaldehyde loaded onto the CPGF NPs was evaluated by TGA. The magnetic property of samples was analyzed using a Physical Property Measurement System (PPMS) from Quantum Design Inc., San Diego, California equipped with a 9 Tesla superconducting magnet. Magnetizations versus magnetic field (M–H) measurements were performed by a VSM attachment by using accurate amount of the samples packed inside a plastic sample holder. M–H loops were recorded at a rate of 75 Oe/s in a field sweep from − 10 to 10 kOe at the vibrating frequency of 40 Hz at 300 K. Radiofrequency absorption was carried out with a 20-MHz oscillator at a fixed nominal power of 100 W.

### Colloidal stability

The colloidal stability of NPs was analyzed by measuring UV-VIS absorbance. All the NPs of 100 µg/ml concentration were taken either in distilled water (DW) or in phosphate buffer saline (PBS) or in cell culture medium DMEM with or without 10% FBS [22]. Stability of NPs was determined by measuring the absorbance of each solution at 540 nm, as a function of time (t).

### Drug release

As-prepared CPGF NPs (50 mg) were put into a 12 kDa cut-off dialysis bag (Sigma-Aldrich, St. Louis, MO, USA) which was immersed into 100 ml of 50 mM sodium acetate buffer having either pH 5.2 or pH 7.4. The whole assembly was stirred for 24 h. The drug release was measured by taking out 1 ml solution at regular intervals of 1, 2, 4 and 24 h and analyzed for UV-VIS absorbance [23] at 290 nm, the absorbance maximum of cinnamaldehyde [24].

### Biocompatibility

The Institutional Ethical Committee Bharati Vidyapeeth University Medical College specifically approved this study. Fresh human whole blood (5 ml) was obtained from a healthy donor and centrifuged at 1000 rpm for 15 min to separate RBCs that were washed with saline and diluted to 1∶4 ratio. Saline was used as a negative control and distilled water was used as a positive control. Different concentrations of CPGF NPs (0.5, 1, 5 and 10 mg/ml) were mixed with 1∶4 diluted blood sample and incubated at 37°C for 30 min. The tubes were centrifuged at 3000 rpm for 5 min, the supernatant was collected and optical density (OD) was determined at 545 nm. The hemolysis rate (HR) was calculated using the mean OD for each group as follows:


The samples were referred [25] to be highly hemocompatibile for HR <5%, hemocompatible for HR <10%, and non-hemocompatible for HR>20%. If HR was less than 5%, the sample would have no hemolytic reaction and thus would be considered as hemocompatibile.

### Uptake of CPGF NPs into the breast cancer cells

The internalization of CPGF NPs into the cells was qualitatively evaluated by Prussian blue staining as described previously [26]. MDAMB231 and MCF7 were seeded on coverslips in 6-well plates at a seeding density of 1×10^5^ cells/ml. Next day, the cells were treated with CPGF NPs for 24 h. Post treatment, the cells were fixed with 4% paraformaldehyde for 20 min at room temperature. Cells were washed twice with 1X PBS. The coverslips were immersed in Prussian blue stain which was prepared by mixing equal volumes of 20% aqueous solution of HCl and 10% aqueous solution of potassium ferrocyanide [K_4_Fe(CN)_6_.3H_2_O] for 20 min. The cells were counterstained with neutral red for 5 min. The stained cells were photographed with Sony DSC-S75 cyber-shot camera under 40X objective.

### MTT assay

The effect of CPGF NPs on the viability of MDAMB231, MCF7, MCF10A and HEK 293 was analyzed by using MTT dye [26]. The cells were seeded at 1×10^5^ cells/ml density in 96-well plates (Axygen TPP, CA, USA). After 24 h, the cells were incubated with fresh medium containing different concentrations (0–320 µg/ml) of NPs and the plates were further incubated for 24 h. The MTT solution (5 mg/ml) was added to each well, followed by 4 h incubation at 37°C in 5% CO_2_ incubator. The intensity of colored formazan derivative was determined by measuring optical density (OD) with the ELISA microplate reader (Biorad, Hercules, CA) at 570 nm (OD_570–630__nm_). The cell viability was expressed in terms of percentage as


### Cell growth analysis

Growth kinetics of breast cancer cells was monitored by cell growth assay [27]. MCF7 and MDAMB231 were seeded at a density of 1×10^5^ cells/ml in 24-well plates. Next day, the cells were treated with different concentrations (0–5 µg/ml for MDAMB231 and 0–40 µg/ml for MCF7) of CPGF NPs. The cells were harvested and counted for viability using trypan blue dye exclusion method for 24, 48 and 72 h.

### Soft agar assay

The assay was performed using the method as reported previously [26]. Briefly, 5×10^3^ cells/ml treated with or without different concentrations of CPGF NPs (0–5 µg/ml for MDAMB231 and 0–40 µg/ml for MCF7) were mixed with 0.35% agarose (DNA grade, GIBCO BRL, CA, USA) at 40°C in culture medium. The mixture was poured onto a previously gelled layer of 0.5% agarose in culture medium in 6-well plates and allowed to solidify. After incubation for 10 days in 5% CO_2_ incubator at 37°C, the colonies were counted using an Axiovert 200 M microscope (Carl Zeiss, Germany).

### Wound healing assay

The migration potential of breast cancer cells was analyzed by the wound healing assay [27]. MDAMB231 and MCF7 cells were plated at a seeding density of 5×10^5^ cells/ml in 24-well plates and grown overnight at 37°C in 5% CO_2_ incubator. An artificial wound was made with 10 µl micropipette after 6 h serum starvation in control as well as cells treated with different concentrations of CPGF NPs (0–5 µg/ml for MDAMB231 and 0–40 µg/ml for MCF7). The cells were incubated for 18 h in a humidified chamber at 37°C and 5% CO_2_ atmosphere. Images of migrating cells were obtained by 10X phase objective of an inverted microscope using Sony DSC-S75 cyber-shot camera at 0 and 18 h.

### Gelatin zymography

The gelatin zymography was performed to detect the presence of extracellular MMP-2. The conditioned medium of control as well as cells treated with different concentrations of CPGF NPs (0–5 µg/ml for MDAMB231 and 0–40 µg/ml for MCF7) was collected and concentrated [27] in Centricon YM-30 tubes (Millipore, MA). All the samples, containing equal amount of total proteins, were mixed with sample buffer (2% SDS, 25% glycerol, 0.1% bromophenol blue and 60 mM Tris- HCl pH 6.8). The samples were then diluted again with sample buffer in 1∶2 ratio. Equal volume of the resulting mixture was then loaded onto 7.5% SDS-polyacrylamide gel containing gelatin (0.5 mg/ml). The gel was washed twice with 0.25% Triton X-100 and incubated overnight in incubation buffer (150 mM NaCl, 100 mM CaCl_2_, 50 mM Tris-HCl pH 7.5, 1% Triton X-100, 0.02% NaN_3_) at 37°C. The gel was stained with staining solution (0.1% Coomassie Brilliant blue R-250 in 40% isopropanol) and destained in 7% acetic acid. Gelatinolytic activity was detected as unstained bands against a blue background. The quantitation of bands in control and treated samples was performed by densitometric analysis using Image J gel analysis tool.

### Mitochondrial membrane potential

Both the breast cancer cell lines were seeded at a density of 1×10^5^ cells/ml in a black 96-well plate and incubated at 37°C in a CO_2_ incubator. Next day, the cells were treated with different concentrations of CPGF NPs (0–5 µg/ml for MDAMB231 and 0–40 µg/ml for MCF7) and were incubated in a CO_2_ incubator at 37°C for 24 h. Following day, the medium was removed and the cells were washed with 1X PBS and incubated with 2.5 µg/ml JC-1 staining solution for 1 h in the dark. Fluorescence readings were measured using the Fluostar Omega microplate reader (BMG Labtech) at 520 nm for JC-1 monomers and at 590 nm for JC-1 aggregates.

### Immunoblotting

Protein expression was evaluated by western blotting as reported previously [27]. Briefly, the cells were seeded at a density of 5×10^5^ cells/ml and treated next day with or without different concentrations of CPGF NPs (0–5 µg/ml for MDAMB231 and 0–40 µg/ml for MCF7). The cells were centrifuged and the pellet was resuspended in 80 µl lysis buffer containing 50 mM Tris (pH 7.4), 5 mM EDTA, 0.5% NP40, 50 mM NaF, 1 mM DTT, 0.1 mM PMSF, 0.5 µg/ml leupeptin (Pro-pure Amersco, Solon, USA), 1 µg/ml pepstatin (Amresco, Solon, USA), 150 mM NaCl, 0.5 µg/ml aprotinin (Amersco, Solon, USA) and protease inhibitor cocktail (Roche, Lewes, UK) followed by incubation on ice for 1 h with intermittent mixing. The cell extract was centrifuged for 20 min at 4°C at 12000 rpm to remove the debris. The protein was estimated using Bradford reagent (Biorad Laboratories Inc, CA, USA). Equal amount of protein was loaded onto a 10% SDS-polyacrylamide gel and transferred electrophoretically to Amersham Hybond-P PVDF membrane (GE Healthcare, UK) in sodium phosphate buffer (pH 6.8). The membrane was blocked in 5% BSA in TST and incubated at room temperature for 30 min with rabbit polyclonal primary antibody for VEGF (sc-507) and caspase-3 (sc-7148) whereas mouse monoclonal primary antibody for α- tubulin (sc-5286) (Santacruz, CA, USA), at 1∶500 dilutions. The membrane was washed in TST and incubated with respective secondary IgG HRP conjugate at 1∶2500 dilution. Proteins were visualized using a chemilluminiscence kit (Amersham ECL Advance western blotting detection kit, GE Healthcare, UK) and densitometric analysis was performed on scanned immunoblot images using the ImageJ (NIH, USA) gel analysis tool.

### Statistical analysis

All the experiments were performed in triplicates and repeated thrice. The data has been presented as mean±SD. Statistical analysis was performed with the Graph Pad prism 4 program using one-way ANOVA. The IC_50_ values were calculated by the formula, Y  =  100×A1/(X+A1), where A1  =  IC_50_, Y  =  response (Y = 100% when X = 0) and X  =  inhibitory concentration using KyPlot version 2.0 beta 13 (32 bit). The p values used for comparisons were <0.05.

## Results and Discussion

### Characterization of CPGF NPs

CPGF NPs were characterized by different techniques such as XRD, FTIR, TEM and VSM. Figure 1A indicates powder diffraction patterns of F, GF, PGF and CPGF NPs, which clearly suggest that iron oxide surface was sequentially modified with glycine, pluronic and cinnamaldehyde. These compositions exhibited characteristic magnetite peaks (2θ) at 30.1, 36.2, 42.4, 52.5, 57.5 and 62.2° corresponding to (220), (311), (400), (422), (511) and (440) planes, respectively (JCPDS card no. 01-088-0315), observed for face centered cubic (fcc) lattice structure of iron oxide [26]. It was significant to note that only magnetite phase was formed during the synthesis of all the iron oxide preparations since diffraction peaks corresponding to other phases such as α-Fe_2_O_3_ (hematite) or γ-Fe_2_O_3_ (maghamite) were found to be absent. The average crystallite size of all the compositions, as calculated from Scherrer equation, was in the range of 10–20 nm. TEM of CPGF NPs (Figure 1B) showed the particle size to be around 20 nm that had gradually increased from ∼5 nm for bare Fe_3_O_4_ (F) (Figure S1 in File S1) after successive tagging of different moieties onto the NPs. The increase in size of the NPs from F to CPGF corroborated with the observed XRD pattern.

**Figure 1:** Physical characterization of CPGF NPs. (**A**) XRD patterns of F, GF, PGF and CPGF NPs. (**B**) TEM image with SAED of CPGF NPs. (**C**) FTIR patterns of F, GF, PGF and CPGF NPs.

Figure 1C shows the FTIR spectra of F, GF, PGF and CPGF NPs. The basic Fe-O stretch (∼719 cm^−1^) was invariably present in all the compositions, clearly reflecting the capping of organic molecules onto the nanoparticle surface. Upon capping of glycine, a broad peak around 3200 cm^−1^ appeared depicting the presence of hydroxy/amino groups on the surface of Fe_3_O_4_ NPs. A strong absorption at 1600 cm^−1^ in GF originated from carboxyl stretch of glycine moiety. The capping of glycine to Fe_3_O_4_ NPs occurred due to electrostatic interaction between positively charged Fe_3_O_4_ and negatively charged glycine. It was interesting to note that, in PGF, signatures at 3200 cm^−1^ and ∼1600 cm^−1^ persisted even after the addition of pluronic. The presence of these signatures, though with a reduced intensity, indicated the attachment of pluronic to GF through hydrogen bond. The remarkable shift of –C = C– and –C = O signatures from 1696 cm^−1^ and 1634 cm^−1^ in PGF towards higher energy side at 1709 and 1695 cm^−1^, respectively, in CPGF, indicated binding of cinnamaldehyde to PGF. Thus, after binding to the hydrophobic end of pluronic, cinnamaldehyde formed a stable electrostatic interaction as is evident from the near merging of the peaks. The FTIR spectra of glycine (G) (Figure S2 in File S1), pluronic (P) (Figure S3 in File S1) and cinnamaldehyde (C) (Figure S4 in File S1) have been given in supplementary information (File S1). Figure 2 depicts the synthesis of CPGF NPs and their release in breast cancer cell. Pluronic F127 has been known to be a versatile polymer for water dispersibility [28]. F127 consists of a hydrophobic (polypropylene, PPO) chain that electrostatically interacts with the hydrophobic cinnamaldehyde whereas the hydrophilic (polyethylene glycol, PEO) end binds to glycine through electrostatic association between –OH end of F127 and -NH_2_ end of glycine. This generates additional hydrophilicity and stability to the CPGF system.

**Figure 2:** Schematic illustration of synthesis of CPGF NPs and their release in breast cancer cell.

TGA was performed to quantify the amount of different coatings onto the surface of Fe_3_O_4_ NPs. Figure 3A shows the stepwise weight loss for all the NPs. Negligible weight loss of ∼3.8% in F NPs corresponded to the adsorbed moisture between 100 and 200°C. GF NPs showed weight loss of ∼5% starting from 100–300°C that confirmed efficient glycine capping. Due to the addition of pluronic in GF, a two-step weight loss corresponding to ∼9.1% was observed in the temperature range of 150–400°C. A pronounced weight loss of ∼27.2% was observed in CPGF NPs that occurred in three-steps in the temperature range from 100–400°C. It could be due to the removal of glycine, pluronic and cinnamaldehyde successfully from the CPGF NPs. Thus, the amount of cinnamaldehyde loaded onto the Fe_3_O_4_ nanoparticles was found to be about 18.1%.

**Figure 3:** Cinnamaldehyde loading and release profiles along with magnetic behavior of CPGF NPs. (**A**) Thermogravimetric analysis of F, GF, PGF and CPGF NPs. (**B**) Release profile of cinnamaldehyde from CPGF NPs at different pH values at different time points. (**C**) Inset shows uniform suspension of CPGF NPs (i) and (ii) response of the NPs to the externally placed magnet. VSM data shows the magnetic behavior of all the NPs.

Figure 3B shows release kinetics of cinnamaldehyde in sodium acetate buffer at pH 5.2 and 7.4 that was analyzed by UV-vis spectroscopy. The drug release kinetics of the NPs was studied to analyze the fate of cinnamaldehyde in a) acidic pH, usually present in the tumor microenvironment and b) physiological pH, corresponding to the body fluids [29]. At both pH values, CPGF NPs showed a short burst release of cinnamaldehyde during initial 4 h, followed by a sustained release profile with increased time periods. Due to electrostatic interaction of cinnamaldehyde with PGF system, it could get easily detached from the CPGF NPs resulting into faster release. The rate of release was found to be slightly more at lower pH that could be attributed to ionic interaction of free aldehyde group of cinnamaldehyde with the liberated protons under acidic conditions. The higher rate of payload release in acidic pH is a good indicator of the efficacy of the system to deliver the drug at the tumor site.

The inset of Figure 3C shows uniform suspension of CPGF NPs (i); upon exposure to the external magnet, the NPs got attracted towards the side of the glass vial, leaving behind a clear suspension (ii). Upon removal of the magnetic field, the NPs got re-dispersed into the clear solution, suggesting their magnetic nature. The magnetic properties of CPGF NPs were further analyzed by VSM at 300 K.

Figure 3C depicts the hysteresis loops of F, GF, PGF and CPGF NPs showing zero remanence and coercivity, indicating that the nanoparticles were superparamagnetic in nature. The magnetization reached a saturation point at about 10 kOe, which was found to be strongly dependent upon the organic coating. It is well-known that the saturation magnetization (M_S_) decreases with the particle size and also depends on the presence of organic coating on the iron oxide nanoparticles [30]. The M_S_ value of F NPs was found to be 59.12 emu/g which was less than the reported value of bulk magnetite (92 emu/g) and could be attributed to the small particle size [31]. The M_S_ value was found to decrease from 59.12 emu/g to 50.97 emu/g (CPGF NPs) with the increase in coatings onto the magnetic core. The NPs capped with glycine (GF) had MS value of 55.7 emu/g that further decreased to 53.99 emu/g with an addition of pluronic (PGF) on it. This decrease in the M_S_ value could be attributed to the presence of non-magnetic coatings onto the surface of Fe_3_O_4_ NPs. The role of glycine and cinnamaldehyde coating was significant as the decrease in M_S_ value for these two materials was almost similar. Interestingly, after addition of pluronic, there was no significant difference in M_S_ value, implying that it played a major role in conjugation of cinnamaldehyde with glycine capped iron oxide NPs.

### Stability and biocompatibility studies

Stability and biocompatibility of the NPs are important pre-requisites for their application in biological domain. The agglomeration of the NPs was examined in different fluids such as DW, PBS, FBS and DMEM (with or without FBS) by measuring their turbidity at 540 nm (Figure 4A). CPGF NPs showed excellent hydrophilicity and were stable in all the tested solutions for 2 h. Interestingly, the NPs showed high colloidal stability in FBS and DMEM supplemented with FBS (Figure 4A) that could be attributed to the adsorption of negatively charged serum proteins onto the Fe_3_O_4_ core. The NPs were found to be biocompatible with no detectable hemolysis activity (<5%) at concentrations ranging from 0.5–10 mg/ml. Hemolysis rates at 0.5, 1, 5 and 10 mg/ml concentrations of CPGF NPs were found to be 3.36, 3.46, 3.57 and 4.64%, respectively, compared to the DW positive control (100%) and saline negative control (2.91%) (Figure 4B). The uptake of CPGF NPs in the breast cancer cells has been shown in Figure 4C. The blue coloured cytoplasm indicated the presence of Fe^3+^ inside the cells (observed at 40X magnification) whereas the untreated control cells, having no NPs, appeared orange-red in colour. Thus, CPGF NPs depicted a highly stable and biocompatible system.

**Figure 4:** Stability, biocompatibility and uptake of CPGF NPs. (**A**) Stability of CPGF NPs in different solutions was monitored by UV-vis spectroscopy. The data is presented as mean±SD of three independent experiments at p<0.0001, indicating statistically significant differences between different solutions. (**B**) Biocompatibility of CPGF NPs performed in freshly prepared human blood. DW and saline were used as positive and negative controls, respectively. The data is presented as mean±SD of three independent experiments at p<0.001, indicating statistically significant differences compared to positive control group. (**C**) In vitro uptake of CPGF NPs in MDAMB231 and MCF7, shown by Prussian blue staining, and compared with their respective untreated control cells. The stained cells were photographed with Sony DSC-S75 cyber-shot camera.

### Growth kinetics of breast cancer cells treated with CPGF NPs

To evaluate whether CPGF system enhanced the bioavailability of cinnamaldehyde in the cancer cells, cytotoxicity assays of the NPs (Figure 5A) as well as F, G and P (Figure S5 in File S1) at different concentrations (0–640 µg/ml), were performed in breast cancer cell lines (MDAMB231 and MCF7). F, G and P were found to be non-toxic to the breast cancer cells (Figure S5 in File S1). However, CPGF NPs (Figure 5A) were found to significantly decrease (p<0.0001) the survival of breast cancer cells from 10 and 80 µg/ml concentrations (corresponding to ∼0.014 and 0.1 µM concentrations of the cinnamaldehyde, respectively, loaded onto the NPs) in MDAMB231 and MCF7, respectively. Interestingly, the NPs were not toxic to the non-cancerous MCF10A and HEK 293 cells upto 640 µg/ml (containing ∼0.9 µM of cinnamaldehyde) (Figure 5A). On the other hand, upon treatment of the cells with different concentrations (0–160 µM) of free cinnamaldehyde (Figure 5B), it induced killing from 40 and 80 µM concentration onwards in MDAMB231 and MCF7, respectively. Such higher concentrations of cinnamaldehyde were also deleterious to the non-cancerous cells, MCF10A and HEK 293. Thus, free cinnamaldehyde was toxic to both the breast cancer as well as the non-cancerous cells at higher doses. However, upon tagging with magnetic nanoparticles, the therapeutic index of cinnamaldehyde was drastically reduced reflecting its increased bioavailability. In MDAMB231 and MCF7 cells, CPGF NPs exhibited IC_50_ of 0.363 and 0.368 µM, respectively (Table S1 in File S1). On the other hand, the free cinnamaldehyde exhibited IC_50_ of 69.81 and 284.7 µM for MDAMB231 and MCF7, respectively. These findings clearly demonstrate that functionalization of MNPs with cinnamaldehyde increased its bioavailability at lower doses, thereby increasing its therapeutic efficacy.

**Figure 5:** Cytotoxicity analysis of CPGF NPs and cinnamaldehyde. The breast cancer (MDAMB231 and MCF7) and non-cancerous (MCF10A and HEK293) cells were treated with different concentrations of (**A**) CPGF NPs and (**B**) cinnamaldehyde for 24 h and anlayzed for viability by MTT assay. Lower panel of X-axis in (**A**) refers to amount of cinnamaldehyde (µM) present in the corresponding concentrations of CPGF NPs (µg/ml) (as calculated from TGA data). All the data are presented as mean±SD of five independent experiments at p<0.0001, indicating statistically significant differences compared to the control untreated group.

The novelty of CPGF nanoparticulate system was that it exhibited cytotoxicity in both ER/PR positive/Her2 negative (MCF7) and ER/PR negative/Her2 negative (MDAMB231) breast cancer cells, the latter being insensitive to most of the chemotherapeutic drugs [32]. The triple-negative breast cancers (ER/PR^−^ Her2^−^) have a more aggressive clinical course than other forms of breast cancer [33]. The lack of ER and PR receptor expression in breast cancer is usually associated with increased visceral metastases, poor prognosis [34], [35], [36], [37] and relatively short relapse-free and overall survival times [33], [38], [39].Interestingly, compared to MCF7 cells, MDAMB231 showed susceptibility to killing by the NPs at much lower doses (low MIC values) of cinnamaldehyde. It has been reported earlier that 2′-benzoyloxycinnamaldehyde (BCA), a derivative of 2′-hydroxycinnamaldehyde, showed more effective antiproliferation in MDAMB231 than in MCF7 due to increase in the expression of DJ-1 protein in the latter [40]. This protein is known to protect the cancer cells from oxidative stress *via* translocalizing into mitochondria and stabilizing mitochondrial permeability and thus increase in its expression in MCF7 cells could explain their resistance to BCA treatment. The same reason could explain the observed difference in sensitivity of MCF7 and MDAMB231 towards CPGF NPs.

Based on the cytotoxicity data, we used non-killing doses of CPGF NPs, (0–10 µg/ml for MDAMB231 and 0–40 µg/ml for MCF7) for further biological assays. The effect of different concentrations of CPGF NPs was analyzed on the growth of breast cancer cells for 24–72 h. Figure 6A shows a dose-dependent decrease in the growth kinetics of MDAMB231 and MCF7 cells (p<0.0001) at 24–72 h. This was supported by a dose-dependent decrease in the number of soft agar colonies in both the cell lines (Figure 6B). Thus CPGF NPs significantly restricted the growth of breast cancer cells in vitro.

**Figure 6:** CPGF NPs decrease the growth kinetics of breast cancer cells. (**A**) The NPs decreased the number of cells in MDAMB231 and MCF7, indicated by cell growth assay. Cells were counted from the four quadrants and the average of each has been plotted. The data represents mean±SD of three independent experiments at p<0.0001 indicating statistically significant differences compared to the control untreated group. (**B**) Reduction in the number of soft agar colonies was observed in MDAMB231 and MCF7 after treatment with CPGF NPs. Colonies were counted from at least 10 different areas and the average of each has been plotted. The data represents mean±SD of three independent experiments at p<0.0001 indicating statistically significant differences compared to the control untreated group.

### Mechanism of anticancer potential of CPGF NPs

Cinnamaldehyde has been reported to control various processes involved in the malignant transformation of cells, such as cell proliferation, invasion and migration that are the key steps in metastasis, one of the major causes of mortality in cancer [41]. To examine the effect of CPGF NPs on cell migration, we performed wound healing assay on confluent monolayers of breast cancer cell lines (Figure 7A). After 18 h, the untreated control cells covered up ∼85% of the wound, whereas at 5 and 40 µg/ml concentrations of CPGF NPs, MDAMB231 and MCF7 cells covered up the wound by ∼47 and 32%, respectively (p = 0.0005) (Figure 7A, B). Thus, the NPs were found to decrease the migration of breast cancer cells in a dose- and time-dependent manner.

**Figure 7:** Molecular mechanism underlying anticancer activity of CPGF NPs. CPGF NPs decreased migration and expression of tumor marker proteins in breast cancer cells. (**A**) The NPs reduced migration of MDAMB231 and MCF7 cells. The upper panel of each figure shows the wound made at 0 h and the lower panel shows the migration of cells after 18 h. (**B**) Graphical representation of wound closure in MDAMB231 and MCF7 at 18 h after CPGF NPs treatment. Values are represented as mean±SD of three independent experiments at p<0.01 for MDAMB231 and p<0.0005 for MCF7, indicating statistically significant differences compared to the untreated control cells. (**C**) Gelatin zymography shows downregulation of MMP-2 expression in MDAMB231 and MCF7 after treatment with CPGF NPs with their corresponding densitometric analysis. The values are represented as mean±SD of three independent experiments at p<0.001, indicating statistically significant differences compared to the untreated control cells. (**D**) Western blot analysis shows decrease in VEGF expression in MDAMB231 and MCF7 with their corresponding densitometric analysis. Values are represented as mean±SD of three independent experiments with p<0.0001, indicating statistically significant differences compared to the untreated control cells.

MMPs, a family of zinc and calcium-dependent enzymes, are known to degrade extracellular matrix proteins resulting into basement membrane degradation that ultimately leads to metastasis [42]. Since MMP-2 significantly contributes towards the invasive property of the cancer cells, we evaluated its expression in the cells treated with CPGF NPs. The expression of MMP-2 was found to be significantly down-regulated (p≤0.001) in both MDAMB231 and MCF7 (Figure 7C), thereby suggesting that the NPs inhibited the migration of breast cancer cells through reduction in MMP-2 expression.

VEGF, an oncoprotein responsible for angiogenesis in cancer cells, plays an important role in tumor metastasis by mediating the formation of lymphatic vessels [43]. VEGF and MMP2 proteins have been reported to be positively correlated with each other in various cancers, including breast cancer and have been proposed to be potential tumor markers [44]. VEGF has been known to not only stimulate the proliferation and migration of endothelial cells, but also to activate the inactive pro-MMPs to active MMPs [45]. The latter in turn degrade the vascular basal membrane and ECM proteins, resulting into the migration of endothelial cells and formation of new blood vessels [42]. We found that CPGF NPs significantly down-regulated (p<0.0001) the expression of VEGF in both the breast cancer cell lines in a dose-dependent manner compared to the untreated control cells (Figure 7D).

Cinnamaldehyde has been reported to induce apoptosis via caspase-3 activation. Since CPGF NPs altered the growth kinetics of breast cancer cells, we examined the effect of CPGF NPs on the mitochondrial membrane potential of both the breast cancer cell lines. Interestingly, CPGF NPs treatment resulted into the disruption of the mitochondrial membrane potential (Dym) that was observed by a dose-dependent decrease (p<0.0001) in red fluorescence intensity, after staining the cells with JC-1 dye (Figure 8A). This was supported by a corresponding increase (p<0.0001) in the expression of caspase-3 in cells treated with CPGF NPs as compared to the untreated control cells (Figure 8B). The loss of mitochondrial membrane potential is the hallmark of apoptosis. These results indicated that cinnamaldehyde-Fe_3_O_4_ induced apoptosis in breast cancer cells through mitochondria dependent pathway.

**Figure 8:** CPGF NPs induce apoptosis in breast cancer cells. (**A**) CPGF NPs decreased the mitochondrial membrane potential of the breast cancer cell lines as observed by JC-1 staining. The data was analyzed by the MARS data analysis software 2.10R3 (BMG Labtech). All data are presented as means±SD of three independent experiments. p<0.0001 indicate statistically significant differences compared to the control untreated group. (**B**) Western blot data shows increase in caspase-3 expressions in both MDAMB231 and MCF7. α-Tubulin was used as a loading control. The histogram depicts densitometric analysis of western blots of caspase-3. Values are represented as mean±SD of three independent experiments. p<0.001 indicate statistically significant differences compared to the untreated control cells.

The mechanistic studies confirmed the potential of CPGF NPs to restrict the growth of breast cancer cells through inhibition of migration, invasion and induction of apoptosis. Therefore, PF127-Glycine-Fe_3_O_4_ could be an appropriate carrier for hydrophobic agents such as cinnamaldehyde to improve their bioavailability in cancer therapy.

### Hyperthermia potential of CPGF NPs

Iron oxide nanoparticles have been used in hyperthermia [46] because of their ability to get heated upto 42–45°C upon exposure to radiation. The magnetite NPs tagged with different anticancer drugs such as doxorubicin [18] or anti-Her2 immunoliposomes [19] have been extensively explored for targeted delivery and hyperthermia in breast cancer. Since CPGF NPs showed enhanced anticancer activity in both ER/PR positive/Her2 negative (MCF7) and ER/PR negative/Her2 negative (MDAMB231) breast cancer cells, we wanted to know whether the NPs had the potential for application in cancer hyperthermia as well. Thus, solutions (10 mg/ml) of F, G, P, C and CPGF NPs in deionized water, were subjected to 20 MHz RF radiation [47] for different time periods (0–150 s), and the temperature rise was monitored (Figure 9). CPGF NPs showed a significant rise in the temperature to 41.6°C within a time span of 1 min. Such rise in temperature upon RF exposure has been reported to be dependent upon the magnetic nature, polar/non-polar nature as well as the concentration of the nanoparticles [48], [49]. The results appeared to be quite encouraging since the tumors get ablated at 41.6°C while the normal cells are known to withstand higher temperatures [50].

**Figure 9:** Response of CPGF NPs to the radiofrequency waves for hyperthermia application. CPGF NPs exhibit hyperthermia potential. Response of Fe_3_O_4_ (F), Glycine (G), Pluronic (P), Cinnamaldehyde (C) and CPGF NPs to the radiofrequency waves have been depicted. The NPs showed a significant rise in the temperature to 41.6°C within a time span of 1 min.

## Conclusions

In summary, cinnamaldehyde, a natural anticancer hydrophobic compound present in *Cinnamomum* sp, was tagged with PF127-Glycine-Fe_3_O_4_ system that increased its bioavailability and in turn its therapeutic efficacy in breast cancer cells. The resulting CPGF NPs served as a vehicle for targeted delivery of cinnamaldehyde and exhibited anticancer and hyperthermia potential in breast cancer.

## Supporting Information

File S1 **Supporting Information that includes Table S1, Table S2, and Figure S1 - Figure S5.** Cytotoxic studies of cinnamaldehyde and its derivatives (Table S1) as well as those of MNPs loaded with herbal active compounds (Table S2). Physical characterization of F, G, C, P, GF, PGF and CPGF NPs (Figures S1–S4) and cytotoxicity data of F, G and P (Figure S5). Table S1. Cytotoxic studies of cinnamaldehyde and its derivatives. Table S2. Cytotoxic studies of MNPs loaded with herbal active compounds. Figure S1. TEM images of F, GF and PGF NPs. TEM image showed the particle size to be around 5–10 nm for F and GF NPs and ∼10–15 nm for PGF NPs. This indicated that the size of the NPs gradually increased from ∼5 nm for non-conjugated Fe_3_O_4_ to ∼20 nm for PGF NPs by successive layering of G and P onto the F NPs. Figure S2. FTIR spectra of F, G and GF. Glycine spectrum (G) showed remarkable signatures at ∼3200 cm^−1^ for −NH_2_ or −OH and that for carboxylate stretch at ∼1600 cm^−1^. The notable difference between Fe_3_O_4_ spectrum (F) and glycine capped Fe_3_O_4_ (GF), was the appearance of a strong new signature at 3200 cm^−1^, along with 1600 cm^−1^. This indicated that Fe_3_O_4_ surface was efficiently capped with glycine. Figure S3. FTIR spectra of GF, P and PGF. The appearance of peaks at 3200 cm^−1^ and 1600 cm^−1^ (1696 cm^−1^ in PGF) for both GF and PGF suggested that the hydroxyl/amine and carboxylate functions of G and P are successively loaded onto the Fe_3_O_4_ NPs. The overall merging of peaks indicated that pluronic possessed similar functional groups as in glycine resulting in similar spectrum of PGF to GF. Figure S4. FTIR spectra of PGF, C and CPGF. Cinnamaldehyde spectrum (C) showed prominent peaks at 1696, 1634, 1140, 960 and 764 cm^−1^ arising due to bonds specified by aldehyde structure. There was an interesting shift of –C = C– and –C = O stretches from 1696 and 1634 cm^−1^ in PGF towards higher energy side at 1709 and 1695 cm^−1^ in CPGF denoting conjugation of cinnamaldehyde with PGF. The invariable presence of other peaks in cinnamaldehyde such as 1140, 960 and 764 cm^−1^ in CPGF spectrum suggested that cinnamaldehyde was electrostatically bound to PGF. Figure S5. Cytotoxicity of F, G and P. The effect of F, G and P on MDAMB231 and MCF7 was analyzed by using MTT dye. The cells were treated with 0–640 µg/ml of F, G and P. Uncoated Fe_3_O_4_ nanoparticles were non-toxic to all the cell lines which is in accordance with the previously reported data. Both the cell lines showed ≥100% viability post-treatment with glycine and pluronic used to coat Fe_3_O_4_ nanoparticles. Therefore, these coating materials were non-toxic and safe.
(DOCX)
